# Influenza A Virus Production in Mouse Lung Is Inhibited by Inhalation of Aerosol Polyethylenimine/Short Hairpin RNA Plasmid Complexes

This article has been retracted.

**DOI:** 10.1155/2022/7404813

**Published:** 2022-04-22

**Authors:** Liang Shi, Shenhui Yin, Hao Ren, Rong Gao, Zhuang Ma, Wenwu Sun, Jianping Cao

**Affiliations:** ^1^Department of Respiratory and Critical Care Medicine, General Hospital of Northern Theater Command, Shenyang 110016, China; ^2^Department of Naval Medicine, Naval Medical University, Shanghai 200433, China

## Abstract

Influenza pandemics are a global threat to human health, with existing vaccines and antiviral drugs providing limited protection. There is an urgent need for new prophylactic and treatment strategies. In this study, 12 short hairpin (sh)RNAs targeting conserved regions of influenza A virus (IAV) matrix protein (M)2, nucleocapsid protein (NP), nonstructural protein (NS), and polymerase acidic (PA) were synthesized, and their effects on IAV replication in cells were investigated using Madin–Darby canine kidney (MDCK) cells transfected with the shRNA plasmids. Additionally, mice were administered a polyethyleneimine PEI/pLKD-NP-391 complex in aerosol form and then infected with AIV, and viral particles in the mouse lung were detected. IAV production was markedly lower in MDCK cells transfected with pLKD-M-121, pLKD-M-935, pLKD-NP-391, pLKD-NP-1291, pLKD-PA-1365, and pLKD-PA-1645 plasmids than in control cells (*p* < 0.01). The viral load in MDCK cells was decreased by transfection of plasmids pLKD-M-121 (*p* < 0.05) and pLKD-M-935, pLKD-NP-391, pLKD-NP-1291, pLKD-PA-1365, and pLKD PA-1645 (*p* < 0.01) compared to an empty plasmid. The viral load was significantly lower in the lungs of mice transfected with pLKD-NP-391 than in the control plasmid and mock transfection groups (*p* < 0.01 and *p* < 0.05, respectively). Thus, IAV production was inhibited by shRNAs targeting matrix IAV components; moreover, inhalation of a PEI/pLKD-NP-391 complex in aerosol form suppressed IAV production in infected mice. Thus, these shRNAs can be effective for the prevention and treatment of influenza virus infection.

## 1. Introduction

Influenza A virus (IAV) infection is a major public health concern because of its high pathogenicity in patients and the high mortality from viral pneumonia. IAV is characterized by aggregation and high infectivity, and infections have an acute onset and progress rapidly [1]. Traditional antiviral drugs have low efficacy as the virus exists inside cells and because of the emergence of drug-resistant variants; moreover, they have severe side effects that limit their application. Vaccination is a prophylactic measure for IAV infection, but frequent changes in viral antigen (i.e., antigenic drift) render previous vaccines ineffective. Meanwhile, the development of new vaccines lags behind the spread of new variants [2].

RNA interference (RNAi), in which double-stranded RNA directs sequence-specific degradation of homologous mRNA [3–5], has the potential to overcome the abovementioned problems. Small interfering (si)RNAs targeting conserved regions of the influenza virus genome can potently inhibit virus production in cell lines [6] and were shown to be effective in preventing and treating influenza virus infection in mice [7]. Additionally, siRNAs specific for matrix protein (M)2 and nucleocapsid protein (NP) of the H5N1 strain inhibited the replication of different IAV subtypes (H5N1, H7N9, and H1N1) [8].

The IAV genome consists of 8 RNA segments; 2 of these are hemagglutinin and neuraminidase, which undergo frequent antigenic drift and are thus unsuitable RNAi targets. The other 6 segments are essential for virus replication and are conserved across virus subtypes. In the present study, we designed 12 short hairpin (sh)RNA targeting IAV M2, NP, nonstructural protein (NS), and PA and investigated their effects on IAV production in infected cells and in mice.

## 2. Methods

### 2.1. Virus, Cells, and Animals

IAV A/Shanghai/N33/(2008) H1N1 and Madin–Darby canine kidney (MDCK) cells were provided by the Department of Naval Medicine, Naval Military Medical University. All experiments with H1N1 were conducted in an animal biosafety level 3 laboratory at Naval Military Medical University. MDCK cells were cultured in Dulbecco's Modified Eagle's Medium (DMEM) containing 10% fetal calf serum (FCS), 2 mM l-glutamine, 100 U/ml penicillin, and 100 *μ*g/ml streptomycin at 37°C and 5% CO_2_. Female BALB/c mice aged 5 to 6 weeks were purchased from Animal Center of Naval Military Medical University. The animals had free access to food and water throughout the study. All animal procedures were approved by the Committee on Ethics of Biomedicine, Naval Military Medical University.

### 2.2. shRNA and Plasmid Construction

Four RNA fragments of strain H1N1 (M2, NP, NS, and PA) were transcribed into cDNAs, which were sequenced by Shenggong Biotechnology Co. (Shanghai, China). Three pairs of shRNAs were designed against each fragment, and the 12 pairs of oligonucleotides plus 1 pair of a scrambled oligonucleotide that served as a negative control were synthesized by Obio Technology Co (Shanghai, China). The shRNA expression plasmid pLKD-CMV-G&PR-U6-shRNA was provided by Obio Technology Co.; the sequences of all tested shRNAs are shown in Table 1. The 13 pairs of oligonucleotides were annealed and inserted into the *Age*I and *Eco*RI sites of the shRNA expression vector pLKD-CMV-G&PR-U6-shRNA harboring ampicillin and puromycin resistance genes. The shRNA plasmid used for mock transfection (pLKD-007) encoded a hairpin shRNA whose sequence was not found in mouse, human, or IAV genomes. The recombinant plasmids were transformed to *Escherichia coli*, and positive clones were selected by PCR amplification using the following primers: 5′-TACGATACAAGGCTGTTAGAGAG-3′ (forward) and 5′-CTATTAATAACTAATGCATGGC-3′ (reverse). The forward and reverse primers targeted a sequence of the human U6 promoter and the 5′ sequence of the cytomegalovirus (CMV) promoter, respectively Table 2. Positive clones were confirmed by sequencing.

### 2.3. Plasmid Transfection

MDCK cells were cultured in DMEM containing 10% FCS, 2 mM l-glutamine, 100 U/ml penicillin, and 100 *μ*g/ml streptomycin at 37°C and 5% CO_2_. For shRNA transfection, cells in log growth phase were seeded in a 24-well plate at 5 × 10^4^/well. When the cell layer reached 70%–80% confluence, they were transfected with the plasmids using Lipofectamine 3000 reagent (Invitrogen, Carlsbad, CA, USA) according to the manufacturer's instructions. The plasmid was added to wells of a 24-well plate in triplicate, and the plate was incubated at 37°C and 5% CO_2_; 24 h later, the cells were observed under an epifluorescence microscope to confirm the expression of enhanced green fluorescent protein (eGFP).

### 2.4. Puromycin Screening and Virus Infection

At 24 h after transfection, the culture medium was removed, and cells were washed 3 times with phosphate-buffered saline (PBS) and cultured in influenza virus maintenance medium (DMEM supplemented with 2 mM l-glutamine, 100 U/ml penicillin, 100 *μ*g/ml streptomycin, 0.2% bovine serum albumin, and 25 mM 4-(2-hydroxyethyl)-1-piperazineethanesulfonic acid [HEPES]) containing 2.5 *μ*g/ml puromycin for 48 h to kill untransfected cells. The culture medium was removed, and the cells were washed 3 times with PBS. A 1 ml volume of influenza virus maintenance medium containing 2 *μ*g/ml tosylphenylalanine chloromethyl ketone–trypsin and 5 × 10^7^ 50% tissue culture infective dose (TCID50) H1N1 was added to each well. After 2 h, the culture medium was removed, and the cells were washed 3 times with PBS and cultured in influenza virus maintenance medium at 37°C and 5% CO_2_; 48 h later, the culture supernatant was harvested, and viral load was determined by reverse transcription PCR.

### 2.5. Plasmid Transfection and Virus Infection in Mice

Female BALB/c mice (*N* = 30) were divided into control, mock transfection, and pLKD-NP-391 groups (10 mice each). The pLKD-NP-391 and pLKD-007 plasmids were mixed with polyethylenimine (PEI) (Qbiogene, Carlsbad, CA, USA) at a nitrogen/phosphorus weight ratio of 15 : 1 at room temperature for 20 min [9]. PEI/pLKD-NP-391 or PEI/pLKD-007 was aerosolized using the PARI BOY nebulizer (PARI GmbH, Starnberg, Germany). The aerosol was passed through the sealed plastic cage (12 × 10 × 29 cm) housing the 10 mice. The mice in the treatment groups were administered 2 mg PEI/pLKD-NP-391 or PEI/pLKD-007 in aerosol form for 30 min a day for 3 consecutively days, and control mice were administered the same volume of PBS in aerosol form. At 24 h after the last aerosol administration, the mice were anesthetized with isoflurane followed by intranasal instillation with 50 *μ*l of PBS containing 5 × 10^6^ TCID50 H1N1 virus.

### 2.6. Total RNA Extraction and Quantitative Real-Time (qRT)-PCR

At 48 h after virus infection, mice were sacrificed and homogenates of the right lung lobes were prepared. Total RNA was isolated from the homogenates using TRIzol (Life Technologies, Carlsbad, CA, USA) according to the manufacturer's instructions and stored at −70°C. IAV nucleic acids in the cell culture supernatant were extracted using the PureLink Viral RNA/DNA kit (Life Technologies). Total RNA was reverse transcribed into cDNA using the Prime Script RT Master kit (Takara Bio) at 42°C for 15 min and 95°C for 5 min, and qRT-PCR was performed using the SYBR R Premix Ex Taq kit (Takara Bio, Otsu, Japan) using the following forward and reverse primers: H1N1, 5′-TTCTAACCGAGGTCGAAACG-3′ and 5′-ACAAAGCGTCTACGCTGCAG-3′; and *β*-actin, 5′-AAATCGTGCGTGACATCAAAG-3′ and 5′-AAGAAGGAAGGCTGGAAAAGAG-3′. The annealing temperature was 60°C for both reactions. All reactions were performed in triplicate. The mRNA expression level of IAV in the lung tissue of mice was normalized by subtracting the cycle threshold value of *β*-actin from that of IAV.

### 2.7. Observation of Fluorescence in Frozen Lung Tissue Sections

At 48 h after virus infection, mice were sacrificed and the left lung was dissected. Frozen sections were prepared, and eGFP fluorescence was observed under an epifluorescence microscope.

### 2.8. Statistical Analysis

Data are expressed as mean ± SD. Between-group comparisons were performed with the unpaired Student's *t* test. *p* < 0.05 was considered significant.

## 3. Results

### 3.1. shRNAs Suppress IAV Production in Transfected MDCK Cells

We evaluated the inhibitory effects of shRNAs targeting 4 fragments of IAV (Figures 1(a) and 1(b)) on virus production by transfecting the plasmids harboring the shRNAs into MDCK cells. eGFP expression was detected in the transfected cells (Figure 2). The viral load was significantly reduced in cells transfected with pLKD-M-121, pLKD-M-935, pLKD-NP-391, pLKD-NP-1291, pLKD-PA-1365, and pLKD-PA-1645 compared to those transfected with the control plasmid (*p* < 0.01); it was also lower in cells transfected with pLKD-M-121 (*p* < 0.05) and pLKD-M-935, pLKD-NP-391, pLKD-NP-1291, pLKD-PA-1365, and pLKD-PA-1645 (*p* < 0.01) than in mock-transfected cells. There was no difference in viral load between cells mock-transfected cells and those transfected with the control plasmid (*p* > 0.05) (Figure 3).

### 3.2. Delivery of PEI-pLKD-NP-391 Complexes into the Lungs of H1N1-Infected BALB/c Mice Reduces Virus Production

We investigated whether the shRNAs could reduce the viral load in IAV-infected mice. We selected the shRNA expression plasmid pLKD-NP-391 for the in vivo experiment because it showed the strongest inhibitory effect against the virus in MDCK cells among the tested shRNAs. Mice were administered PEI/pLKD-NP-391 or PEI/pLKD-007 in aerosol form, the left lung was removed, and frozen sections were prepared for analysis of fluorescence under a microscope. The eGFP signal was observed in lung sections of mice transfected with pLKD-NP-391 but not control mice (Figure 4). Moreover, the viral load in the lungs of mice in the pLKD-NP-391 group was significantly lower than that in control and mock-transfected groups (*p* < 0.01 for pLKD-NP-391 vs. control and *p* < 0.05 for pLKD-NP-391 vs. mock-transfected cells). Thus, IAV production in mice was significantly inhibited by the shRNA targeting IAV NP (Figure 5).

## 4. Discussion

siRNAs are an evolutionarily conserved antiviral defense mechanism. Double-stranded RNA with a complementary sequence can degrade endogenous mRNA, resulting in phenotypic aberrations [10]. RNAi targeting viral components involved in gene expression or structural proteins can be exploited for therapeutic purposes; indeed, it was demonstrated that virus infections can be treated by siRNAs [10–12]. In a randomized, double-blind, placebo-controlled trial, the rate of respiratory syncytial virus infection was 44.2% in subjects treated with siRNA compared to 71.4% in those treated with placebo, with no obvious adverse events reported [13]. This was the first application of siRNA as an antiviral agent in humans, and the results were encouraging. The gene silencing effect of the siRNA can be enhanced by modification with PEI to increase biocompatibility [14].

IAV production in infected MDCK cells was suppressed by 6 out of the 12 shRNAs tested; of these, pLKD-NP-391 showed the strongest effect (70% inhibition), followed by pLKD-PA-1365 and pLKD-PA-1645 (65%); only about 37%–50% inhibition was observed with pLKD-M-121, pLKD-M-935, and pLKD-NP-1291. IAV NP and PA play important roles in virus replication. siRNAs targeting these fragments were shown to interfere with the accumulation of not only these transcripts but also of other viral genes including M, NS, PB1, PB2, and PA [6], which is supported by our findings. The authors speculated that siRNA targeting NP caused the degradation of the mRNA, thereby blocking further viral transcription, replication, and new virion production, highlighting the requirement for newly synthesized NP and PA proteins in IAV replication. They also showed that the M protein was not required until a late stage of virus infection. However, an in vitro study showed that an shRNA specific for M2 had a more potent inhibitory effect on H1N1 than one targeting NP, and that NP mRNA accumulation and protein expression were inhibited by an shRNA targeting M2 [15].

Our results showed that the shRNA plasmids were successfully transfected into mice by inhalation of a PEI/plasmid mixture in aerosol form. Because the backbone vector for the shRNAs harbored the eGFP gene, we were able to directly observe green fluorescence in the respiratory tract and pulmonary alveoli in frozen lung tissue sections from the mice. We also demonstrated that viral load in the mice was inhibited by transfection with pLKD-NP-391 but not the control plasmid. This is in agreement with other reports [8, 16], although those studies used an intravenous mode of plasmid delivery. Notably, the PEI/shRNA plasmid mixture was successfully transfected into the lungs of the mice through inhalation of the mixture delivered in aerosol form. This is important for clinical application because the main site of influenza virus infection is the respiratory mucosa including nasal sinuses, bronchiolar epithelium, and alveolar cells; we showed that shRNAs specific for IAV H1N1 can be directly delivered to respiratory epithelial cells targeted by the virus. Moreover, compared to intravenous or intratracheal administration, shRNA delivered in aerosol form has a higher transfection efficiency and uniform distribution in the lungs. Taken together, our preclinical data suggest that shRNAs targeting IAV is a promising prophylactic and therapeutic strategy for influenza that warrant further evaluation in clinical studies. However, our study existed in some limitations. In this study, we used BALB/c mice whose immune system is weak, the effect of this platform on other animal models with robust immune system needs to be investigated in the future. In addition, no side effects of current treatment were reported to date; however, we cannot exclude the possibilities caused by aerosol treatment. Therefore, future studies are also needed to address this issue.

## Figures and Tables

**Figure 1:** Recombinant expression plasmid construction. (a) pLKD-CMV-G&PR-U6-shRNA was digested with *Age*I and *Eco*RI to obtain a 8.2 kb vector fragment and the 312 bp *ccdB* gene. Lane 1, undigested vector; lane 2, vector digested with *Age*I and *Eco*RI; lane 3, DNA ladder marker: 10, 8, 6, 5, 4, 3.5, 3, 2.5, 2, 1.5, and 1 kb and 75, 500, and 250 bp. (b) Transformants were identified by colony PCR. Lane 1, negative control (water); lane 2, negative control (mock plasmid; 586 bp); lane 3, DL2000 DNA marker; lanes 4–11, positive clones (332 bp).

**Figure 2:** eGFP expression of recombinant plasmids in MDCK cells. (a) Cells transfected with mock plasmid. (b) Cells transfected with the pLKD-NP-391.

**Figure 3:** Reduced IAV load in MDCK cells transfected with shRNA expression plasmids. Viral load was decreased in MDCK cells transfected with pLKD-M-121, pLKD-M-935, pLKD-NP-391, pLKD-NP-1291, pLKD-PA-1365, and pLKD-PA-1645 compared to mock-transfected control cells. Data from 2 independent experiments are shown. ^#^*p* < 0.01 vs. control; ∗*p* < 0.05, ∗∗*p* < 0.01 vs. mock plasmid.

**Figure 4:** eGFP expression in the lung of a mouse transfected with pLKD-NP-391 or control vector. (a) Section of control lung tissue. No fluorescence was observed. (b) Section of lung tissue from a mouse transfected with pLKD-NP-391. Green fluorescence was visible in epithelial cells of the bronchiole, terminal bronchiole, and pulmonary alveoli.

**Figure 5:** Inhibition of IAV production by transfection of pLKD-NP-391. Viral load was significantly reduced in the lung of pLKD-NP-391–treated mice compared to the control and mock plasmid-treated mice. ^#^*p* < 0.05 vs. mock plasmid; ∗∗*p* < 0.01 vs. control.

**Table 1:** Sequences of tested small interfering RNAs.

Name	5′	Stem	Loop	Stem	3′
M-121-F	Ccgg	GCTCTCATGGAATGGCTAAAG	CTCGAG	CTTTAGCCATTCCATGAGAGC	TTTTTTg
M-121-R	Aattcaaaaaa	GCTCTCATGGAATGGCTAAAG	CTCGAG	CTTTAGCCATTCCATGAGAGC	
M-548-F	Ccgg	GCACTACAGCTAAGGCTATGG	CTCGAG	CCATAGCCTTAGCTGTAGTGC	TTTTTTg
M-548-R	Aattcaaaaaa	GCACTACAGCTAAGGCTATGG	CTCGAG	CCATAGCCTTAGCTGTAGTGC	
M-935-F	Ccgg	GCTGTGGATGCTGACGATAGT	CTCGAG	ACTATCGTCAGCATCCACAGC	TTTTTTg
M-935-R	Aattcaaaaaa	GCTGTGGATGCTGACGATAGT	CTCGAG	ACTATCGTCAGCATCCACAGC	
NP-391-F	Ccgg	GCTGGTCTGACTCACATAATG	CTCGAG	CATTATGTGAGTCAGACCAGC	TTTTTTg
NP-391-R	Aattcaaaaaa	GCTGGTCTGACTCACATAATG	CTCGAG	CATTATGTGAGTCAGACCAGC	
NP-1034-F	Ccgg	GCTTCATCAGAGGGACAAAGG	CTCGAG	CCTTTGTCCCTCTGATGAAGC	TTTTTTg
NP-1034-R	Aattcaaaaaa	GCTTCATCAGAGGGACAAAGG	CTCGAG	CCTTTGTCCCTCTGATGAAGC	
NP-1291-F	Ccgg	GGGAATGCAGAGGGAAGAACA	CTCGAG	TGTTCTTCCCTCTGCATTCCC	TTTTTTg
NP-1291-R	Aattcaaaaaa	GGGAATGCAGAGGGAAGAACA	CTCGAG	TGTTCTTCCCTCTGCATTCCC	
NS-49-F	Ccgg	GCTTTCAGGTAGATTGCTTTC	CTCGAG	GAAAGCAATCTACCTGAAAGC	
NS-49-R	Aattcaaaaaa	GCTTTCAGGTAGATTGCTTTC	CTCGAG	GAAAGCAATCTACCTGAAAGC	
NS-221-F	Ccgg	GGAGAGGATTCTGAAGGAAGA	CTCGAG	TCTTCCTTCAGAATCCTCTCC	TTTTTTg
NS-221-R	Aattcaaaaaa	GGAGAGGATTCTGAAGGAAGA	CTCGAG	TCTTCCTTCAGAATCCTCTCC	
NS-485-F	Ccgg	GGGAGCAATTGTTGGCGAAAT	CTCGAG	ATTTCGCCAACAATTGCTCCC	TTTTTTg
NS-485-R	Aattcaaaaaa	GGGAGCAATTGTTGGCGAAAT	CTCGAG	ATTTCGCCAACAATTGCTCCC	
PA-900-F	Ccgg	GGGAATACCACTATATGATGC	CTCGAG	GCATCATATAGTGGTATTCCC	TTTTTTg
PA-900-R	Aattcaaaaaa	GGGAATACCACTATATGATGC	CTCGAG	GCATCATATAGTGGTATTCCC	
PA-1365-F	Ccgg	GGAGAAGTACTGTGTTCTTGA	CTCGAG	TCAAGAACACAGTACTTCTCC	TTTTTTg
PA-1365-R	Aattcaaaaaa	GGAGAAGTACTGTGTTCTTGA	CTCGAG	TCAAGAACACAGTACTTCTCC	
PA-1645-F	Ccgg	GGTTCCATTGGGAAGGTATGC	CTCGAG	GCATACCTTCCCAATGGAACC	TTTTTTg
PA-1645-R	Aattcaaaaaa	GGTTCCATTGGGAAGGTATGC	CTCGAG	GCATACCTTCCCAATGGAACC	
Y007-F	Ccgg	TTCTCCGAACGTGTCACGT	TTCAAGAGA	ACGTGACACGTTCGGAGAA	TTTTTTG
Y007-R	Aattcaaaaaa	TTCTCCGAACGTGTCACGT	TCTCTTGAA	ACGTGACACGTTCGGAGAA	

**Table 2:** shRNA plasmids and their targeting fragments and positions.

Code	Targeting fragment and position	Name of shRNA plasmid
1	M-121	pLKD-M-121
2	M-548	pLKD-M-548
3	M-935	pLKD-M935
4	NP-391	pLKD-NP-391
5	NP-1034	pLKD-NP-1034
6	NP-1291	pLKD-NP-1291
7	NS-49	pLKD-NS-49
8	NS-221	pLKD-NS-221
9	NS-485	pLKD-NS-485
10	PA-900	pLKD-PA-900
11	PA-1365	pLKD-PA-1365
12	PA-1645	pLKD-PA-1645
13	Mock plasmid	pLKD-007∗

∗pLKD-007 has a mock shRNA sequence encoding a hairpin siRNA whose sequence was not found in mice, human, and influenza virus genomes. shRNA: short hairpin RNA.

## Data Availability

The authors confirm that the data supporting the findings of this study are available within the article.

## Abbreviations

DMEM: Dulbecco's Modified Eagle's Medium
eGFP: Enhanced green fluorescence protein
FCS: Fetal calf serum
IAV: Influenza A virus
M2: Matrix protein 2
MDCK cell: Madin–Darby canine kidney cell
NP: Nucleocapsid protein
PA: Polymerase acidic
PBS: Phosphate-buffered saline
PEI: Polyethylenimine
qRT-PCR: Quantitative real-time polymerase chain reaction
RNAi: RNA interference
shRNA: Short hairpin RNA
siRNA: Small interfering RNA
TCID50: 50% tissue culture infective dose.
